# Experimental Study of lncRNA RP11-815M8.1 Promoting Osteogenic Differentiation of Human Bone Marrow Mesenchymal Stem Cells

This article has been retracted.

**DOI:** 10.1155/2021/5512370

**Published:** 2021-03-26

**Authors:** Xiang Sun, Junchuan Cao, Jiusong Han, Bo Jia, Jing Wang, Junxiang Lian, Jianwei Gao, Shuguang Liu, Hui Xiao

**Affiliations:** ^1^Department of Oral and Maxillofacial Surgery, Stomatological Hospital, Southern Medical University (Guangdong Provincial Stomatological Hospital), Guangzhou, Guangdong 510280, China; ^2^Department of Stomatology, Chengdu Women's and Children's Hospital, School of Medicine, University of Electronic Science and Technology of China, Chengdu, Sichuan 611731, China; ^3^Department of Orthopedics, Taian City Central Hospital, Taian, Shandong 271000, China; ^4^Department of Orthodontics, Stomatological Hospital, Southern Medical University (Guangdong Provincial Stomatological Hospital), Guangzhou, Guangdong 510280, China

## Abstract

**Objective:**

This study is aimed at investigating the role of long noncoding RNA (lncRNA) RP11-815M8.1 in the osteogenic differentiation of human bone marrow mesenchymal stem cells (hBMSCs).

**Methods:**

RT-PCR was used to detect the expression of lncRNA RP11-815M8.1 before and after osteogenic differentiation of hBMSCs. The lncRNA RP11-815M8.1 in hBMSCs was overexpressed or silenced via lentiviral transfection. The transfection efficiency was detected by RT-PCR, and the proliferation of hBMSCs was determined by CCK-8. After 14 days of osteogenic differentiation of transfected hBMSCs, the expression of osteogenic transcription factors (ALP, OCN, OPN, Runx2, and Osterix) was detected by alizarin red staining and RT-PCR. The mRNAs directly regulated by lncRNA RP11-815M8.1 and targeted miRNAs were analyzed according to the positional relationship between lncRNA and mRNA in the genome and miRanda software.

**Results:**

The expression of lncRNA RP11-815M8.1 enhanced with increasing osteogenic differentiation time of hBMSCs. Two days after the transfection of hBMSCs, lncRNA RP11-815M8.1 expression was significantly increased in the overexpression group and significantly decreased in the knockdown group, compared to control cells. The CCK-8 assay showed that overexpression and knockdown of lncRNA RP11-815M8.1 did not affect the proliferation of hBMSCs. After 14 days of differentiation of hBMSCs, stronger alizarin red staining was observed in the overexpression groups, and the expression of osteogenic transcription factors was increased in the overexpression group compared to the control. In the knockdown group, alizarin red staining and the expression of osteogenic transcription factors were decreased. Bioinformatics analysis showed that lncRNA RP11-815M8.1 was directly associated with one mRNA, 27 interacting miRNAs, and 20 miRNA-targeted mRNAs.

**Conclusion:**

The osteogenic differentiation of hBMSCs can be promoted by lncRNA RP11-815M8.1 in vitro.

## 1. Introduction

The oral and maxillofacial bone structure is an important basis to support the face, and the repair of maxillofacial bone tissue defects, caused by trauma, tumors, and congenital deformity, is an urgent and difficult issue in oral and maxillofacial surgery [1]. The conventional repair methods like autologous and allogeneic bone grafts have their own disadvantages, for example, the source of autogenous bone is limited and the immune rejection of allogeneic bone was large [2]. However, the recent development of bone tissue engineering has opened up a new opportunity for bone defect repair. The repair process of bone defect includes changes in the balance between osteoclasts and osteoblasts, decreased bone resorption by osteoclasts, concurrent osteoblast chemotaxis in the defect site, activation and differentiation, and coordination, restoration, and repair of the bone defect site with osteoblasts, which mainly originate from bone marrow mesenchymal stem cells (BMSCs) [3, 4]. Human BMSCs (hBMSCs), as important seed cells in bone tissue engineering, have high self-renewal and multidirectional differentiation potential and can be differentiated into osteoblasts under appropriate conditions [5]. Other advantages of hBMSCs include convenient sources, limited damage to the body, and minimized immune rejection after transplantation [6]. Therefore, the mechanism investigation of osteogenic differentiation of hBMSCs will contribute to the clinical application of hBMSCs in bone tissue engineering.

Long noncoding RNAs (lncRNAs) are a series of RNA molecules longer than 200 nucleotides that are not translated into proteins and were initially considered byproducts of the transcription process with no biological function [7]. It has been reported that the complex network regulated by lncRNAs plays an important role in the process of cell and tissue differentiation. For example, studies have shown that lncRNAs are related to differentiation of neuronal [8], muscle [9], epidermal [10], and adipogenic [11]. Recent studies have also found that lncRNAs are involved in the regulation of osteoblastic differentiation of mesenchymal stem cells (MSCs) [12, 13]. However, the potential functions and regulatory mechanisms of lncRNAs in the osteogenic differentiation of hBMSCs remain unclear.

In a previous study using high-throughput sequencing of lncRNAs, we found that lncRNA RP11-815M8.1 was differentially expressed in the osteogenic differentiation process of hBMSCs. This study was conducted to explore the role of lncRNA RP11-815M8.1 in the process of osteogenic differentiation of hBMSCs by RT-PCR detection and lentiviral vector transfection and predict the potential targets of lncRNA RP11-815M8.1 by bioinformatics analysis. Thus, this study provides a new lncRNA target in the mechanism of osteogenic differentiation of hBMSCs and a new strategy for the construction of improved tissue-engineered bone grafts.

## 2. Materials and Methods

### 2.1. Cell Culture and Osteogenic Differentiation

Frozen primary hBMSCs (ScienCell-7500, USA) were placed in a water bath at 37°C until completely thawed and seeded at a density of 5 × 10^3^/cm^2^ in a T-75 culture flask coated with polylysine. Cells were cultured in mesenchymal stem cell growth medium (ScienCell-7501, USA) and incubated at 37°C with 5% CO_2_ and 95% relative humidity. The next day, the medium was changed to remove residual DMSO and the nonadherent cells. After that, the medium was changed every 3 days. When the cells reached 90% confluence, they were trypsinized with 0.25% trypsin/0.02% EDTA, and subculturing was carried out to generate P3 cells. P3 hBMSCs were seeded in 6-well plates at a density of 2 × 10^4^/cm^2^ per well. When the confluence was over 80%, the medium was replaced with MSC osteogenic differentiation medium (ScienCell-7531, USA). The medium was completely changed with fresh osteogenic differentiation medium every 3 days, and the cells were harvested and collected after 7, 14, and 21 days of osteogenic differentiation. RNA was extracted, and the expression of lncRNA RP11-815M8.1 was detected by RT-PCR.

### 2.2. Cell Transfection

The full-length sequence of lncRNA RP11-815M8.1 was obtained from the NCBI database (Table 1). The lncRNA RP11-815M8.1-overexpressing lentiviral vector (OE-RP11-815M8.1) was constructed with the pBABE vector, and the lncRNA RP11-815M8.1-knockdown lentiviral vector (sh-RP11-815M8.1) was constructed with the PLKO.1 vector. All of the above viral vectors were purchased from Anhui General Biotechnology Co., Ltd. Cells at a density of 1.2 × 10^6^ cells/well were seeded in a 6-well plate. After 16 h, the constructed vector was transferred into 293FT cells according to the instruction of the Lipofectamine 2000 (Promega, USA) transfection kit. The medium was changed 8 h after transfection, and the supernatant was collected and stored at 4°C in 48 h. Next, 0.3 mL of the collected supernatant was mixed with MSC culture medium and then added 0.7 mL of cell culture medium and 1.0 *μ*L of polybrene (final concentration was 8 ng/mL). Then, the solution was mixed in hBMSCs cultured Petri dishes with a cell density of less than 60%. One day after MSC culture, the medium was changed to obtain hBMSCs transfected with the lncRNA RP11-815M8.1-overexpressing lentiviral vector (OE-RP11-815M8.1 group), lncRNA RP11-815M8.1-knockdown lentiviral vector (sh-RP11-815M8.1 group), and the corresponding empty transfection vector controls (pBABE group, PLKO.1 group). After 2 days, the cells were collected for extraction of RNA.

### 2.3. CCK-8 Assay

A CCK-8 assay was used to verify the effect of lentiviral vector transfection on the proliferation of hBMSCs. According to the instructions of the CCK-8 Kit (Biyuntian, China), the cells were seeded into 96-well plates at a density of 1 × 10^4^ cells/well, and 10 *μ*L CCK-8 solution was added. The cells were cultured at 37°C, 5% CO_2_, and 95% air humidity. Cell proliferation was detected by the CCK-8 method using a plate reader (Delang, China) at a wavelength of 450 nm on days 2, 5, 8, and 11.

### 2.4. Alkaline Phosphatase (ALP) Staining

The culture medium was removed after osteogenic differentiation; alkaline phosphatase (ALP) staining was performed to identify MSCs according to the instructions of the ALP staining kit (Sigma, USA). The cells were washed twice with phosphate-buffered saline (PBS) and fixed at room temperature with 4% paraformaldehyde for 10 minutes. After fixation, the cells were rinsed again with PBS. An appropriate amount of ALP dye solution was added to the fixed cells in a 6-well plate in the dark and incubated at room temperature for approximately 15-30 minutes. The staining was monitored under a fluorescence microscope every 5 minutes. After the staining was stable, the plate was rinsed with PBS again for final observation. Osteogenic differentiation was confirmed by deepening cytoplasmic staining.

### 2.5. Alizarin Red Staining

To investigate the osteogenic differentiation, alizarin red staining was performed according to the alizarin red kit (Sigma, USA) instruction. The cells were rinsed with PBS and fixed with ethanol for 30 minutes. Next, the liquid was removed, the cells were rinsed twice with PBS, and 2% alizarin red S staining solution was slowly added to the samples, and after incubation at room temperature for 5-10 minutes, the alizarin red solution was removed, after which the cells were rinsed with PBS twice and observed under an inverted microscope. Osteogenic differentiation was validated by increased red calcium salt deposition.

### 2.6. RNA Extraction and RT-PCR Assay

Total RNA was extracted from the cells according to the instructions of the TRIzol Kit (Invitrogen, California, USA) and then reverse transcribed into cDNA using the cDNA reverse transcription kit (TaKaRa, Tokyo, Japan). The cDNA was mixed with the reagents according to the instructions of the SuperReal Fluorescence Quantitative PreMix Color (SYBR Green-FP215) kit (TIANGEN BIOTECH (BEIJING) CO., LTD), and the assay was performed using a real-time quantitative PCR apparatus (Roche LC96, Switzerland). The hBMSCs transfected with the lncRNA RP11-815M8.1-overexpressing lentiviral vector (OE-RP11-815M8.1 group), the RP11-815M8.1-knockdown lentiviral vector (sh-RP11-815M8.1 group), and the corresponding empty control vectors (pBABE group, PLKO.1 group) were incubated with osteogenic induction and differentiation medium for 14 days, and the expression of osteogenic transcription factors (ALP, OCN, OPN, Runx2, and Osterix) was detected by RT-PCR. Osteogenic differentiation was verified by the expression of osteogenic transcription factors. The primer sequences are shown in Table 2.

### 2.7. Prediction of Targeted miRNAs and mRNAs Directly Regulated by lncRNA RP11-815M8.1

According to the positional relationship between lncRNAs and mRNAs in the genome, upstream and downstream transcripts of lncRNAs were found within 100 kb, and these genes and their corresponding transcripts were identified. Since miRNAs play a crucial role in the process of transcriptional regulation, and lncRNAs play an important role in regulating protein-coding genes by binding to miRNAs, the targeting miRNAs of lncRNA RP11-815M8.1 were further predicted by miRanda software.

### 2.8. Statistical Analysis

Statistical graphs were generated by GraphPad Prism 8, and SPSS 22.0 software was used for the statistical analysis. Measurement data are expressed as the mean ± standard deviation. A paired sample *t*-test was used to compare the expression levels between each group and the control group, and *p* < 0.05 indicated a statistically significant difference between groups.

## 3. Results

### 3.1. The Expression of lncRNA RP11-815M8.1 Was Increased during the Osteogenic Differentiation of hBMSCs

After 21 days of osteogenic differentiation of P3 hBMSCs, the cytoplasmic staining was deepened indicating positive ALP staining (Figure 1(a)). Positive alizarin red staining showed red calcium salt deposition (Figure 1(b)). These results indicated the osteogenic differentiation of hBMSCs. The expression of lncRNA RP11-815M8.1 before and after osteogenic differentiation of hBMSCs was detected by RT-PCR, and the results showed that the expression of lncRNA RP11-815M8.1 gradually increased by time (Figure 1(c), Table 3).

### 3.2. Efficiency of Overexpression and Interference of lncRNA RP11-815M8.1 through Lentiviral Vector Transfection and the Effect on hBMSC Proliferation

The lncRNA RP11-815M8.1-overexpressed lentiviral vector, knockdown lentiviral vector, and the corresponding empty vectors were transfected into hBMSCs, and the changes in the expression level of lncRNA RP11-815M8.1 were detected by RT-PCR 2 days later. The results showed that the expression of lncRNA RP11-815M8.1 was significantly increased in the OE-RP11-815M8.1 group (Figure 2(a)) and significantly decreased in the sh-RP11-815M8.1 group compared with the pBABE group and PLKO.1 group (Figure 2(b)), respectively (Table 4).

A CCK-8 assay was used to detect cell proliferation via measurement of cell culture density using a plate reader at the wavelength of 450 nm at 2, 5, 8, and 11 days after hBMSC transfection. The results showed that the overexpression and knockdown of lncRNA RP11-815M8.1 did not affect the proliferation of hBMSCs (Figure 3).

### 3.3. Functional Validation of the Role of lncRNA RP11-815M8.1 in the Process of Osteogenic Differentiation of hBMSCs

The hBMSCs in the OE-RP11-815M8.1 group, the sh-RP11-815M8.1 group, and corresponding control groups (pBABE group, PLKO.1 group) were differentiated in 14 days after induction of osteogenic differentiation, and the effect of osteogenic differentiation was analyzed by alizarin red staining. The results showed that the red calcium salt deposition in the OE-RP11-815M8.1 group was increased compared to the pBABE group. Compared with the PLKO.1 group, the sh-RP11-815M8.1 group had less red calcium salt deposition (Figure 4). The expression of osteogenic transcription factors (ALP, OCN, OPN, Runx2, and Osterix) was detected by RT-PCR, and the results showed that the expression of ALP, OCN, OPN, Runx2, and Osterix increased in the OE-RP11-815M8.1 group in comparison to the pBABE group (Figure 5(a), Table 5). The expression of ALP, OCN, OPN, Runx2, and Osterix in the sh-RP11-815M8.1 group was decreased compared to the PLKO.1 group (Figure 5(b), Table 6).

### 3.4. lncRNA RP11-815M8.1 Directly Regulates mRNAs and Binds to miRNAs

According to the positional relationship between lncRNA and mRNA in the genome, only one mRNA, DUSP10-204, was found within the range of 100 kb upstream and downstream of lncRNA RP11-815M8.1. The targeting miRNAs of lncRNA RP11-815M8.1 were predicted by using miRanda software, and a total of 27 miRNAs related to lncRNA RP11-815M8.1 were found. The mRNAs targeted by the 27 miRNAs were identified in the miRDB database, and 20 of them had score values over 99. The result is shown in Figure 6.

## 4. Discussion and Conclusions

BMSCs have multidirectional differentiation potential and high self-renewal and proliferation abilities. They can differentiate not only into osteoblasts under specific culture conditions *in vitro* but also into osteoblasts *in vivo* by attaching to certain vectors and are considered to be an important choice of seed cells in bone tissue engineering [14]. Therefore, the mechanism investigation of osteogenic differentiation of hBMSCs may contribute to the clinical application in bone tissue engineering.

Initially, lncRNAs were considered to be transcriptional noise of the genome without biological function. However, protein-coding mRNAs account for only 1.5% of RNA transcripts in the mammalian genome; most of the genome consists of noncoding RNAs, such as miRNAs, more than 80% of which are lncRNAs [15]. Studies have shown that lncRNA has a stable secondary structure, different subcellular localization, and higher expression in specific cells and tissues, all of which indicate that lncRNAs are functional [16]. On the other hand, studies in recent years have also found that lncRNAs can regulate gene expression at the epigenetic, transcriptional, and posttranscriptional levels and participate in various essential cellular regulatory processes [17].

Moreover, an increasing number of studies have demonstrated that lncRNAs are closely related to BMSC osteogenic differentiation in recent years. Cao et al. [18] reported that high glucose inhibited the osteogenic differentiation of BMSCs in mice by inhibiting the expression of lncRNA AK028326 and CXCL13. Liang et al. [19] found that miR-141 and miR-22 did target H19 by inducing transcriptional suppression and regulate gene expression in hBMSCs through the classical Wnt/*β*-catenin pathway. Shang et al. [20] showed that TCONS_00041960 regulated osteogenic differentiation of BMSCs in rats by competing as endogenous RNA of miR-204-5p and miR-125a-3p. Wang et al. [21] found that lncRNA MEG3 inhibited the osteogenic differentiation of BMSCs by enhancing the expression of miR-133a-3p and accelerated the occurrence of osteoporosis in postmenopausal osteoporosis patients.

Thus, we screened the differentially expressed lncRNAs before and after osteogenic differentiation of hBMSCs using high-throughput sequencing of lncRNAs in the previous study, including 7 known lncRNAs, 57 unknown lncRNAs, and 409 mRNAs. The lncRNA RP11-815M8.1 was selected due to the large differential expression ratio identified by sequencing experiments, and there has been no research report on its correlation with osteogenic differentiation at present.

We first detected the expression of lncRNA RP11-815M8.1 by RT-PCR before and after 7, 14, and 21 days of osteogenic differentiation of hBMSCs. The results showed that the expression of lncRNA RP11-815M8.1 gradually increased with increasing osteogenic differentiation time suggesting that lncRNA RP11-815M8.1 may promote the osteogenic differentiation of hBMSCs. In this context, lentiviral vectors were used in this study to overexpress and knock down lncRNA RP11-815M8.1 and induced osteogenic differentiation of hBMSCs for 14 days. The results showed that the lncRNA RP11-815M8.1-overexpressing group had increased alizarin red staining and expression of osteogenic transcription factors compared to the control group. The regulation of expression of lncRNA RP11-815M8.1 decreased alizarin red staining and osteogenic transcription factor expression, thus demonstrating that lncRNA RP11-815M8.1 can promote osteogenic differentiation of hBMSCs in vitro.

Cell differentiation can be regulated by lncRNAs via different mechanisms and can play an important role by direct regulation of neighboring protein-coding genes or indirect regulation of protein-coding genes after binding with miRNAs. Based on the positional relationship between lncRNA and mRNA in the genome, we found that the mRNA DUSP10-204 might be directly regulated by lncRNA RP11-815M8.1. The targeting miRNAs of lncRNA RP11-815M8.1 were further predicted by miRanda software, and a total of 27 miRNAs and 20 miRNA-targeted mRNAs were found. The mRNAs which may be directly regulated by lncRNA RP11-815M8.1 could be validated; the effect of binding miRNA to their target genes should be investigated in the future.

This study first revealed the important role of lncRNA RP11-815M8.1 in the process of osteogenic differentiation of hBMSCs and predicted which miRNAs it might bind to and which mRNAs it regulates. This will provide a good preliminary basis for further studies on the mechanism of osteogenic differentiation of hBMSCs. However, no animal model was established in this study, and the function and mechanism of lncRNA RP11-815M8.1 in vivo need to be verified in the future. This will help to reveal a new mechanism of osteogenic differentiation of hbMSCs regulated by specific lncRNA and is expected to improve the efficiency of osteogenic differentiation of hbMSCs, thus providing new ideas and research targets for future bone tissue engineering research.

## Figures and Tables

**Figure 1:** Osteogenic differentiation of hBMSCs: (a) ALP staining; (b) alizarin red staining; (c) changes in the expression level of lncRNA RP11-815M8.1 (^∗∗^*p* < 0.01); the data was normalized to the D0 group which was set as 100%.

**Figure 2:** Transfection efficiency of the overexpression and knockdown of lncRNA RP11-815M8.1. (a) lncRNA RP11-815M8.1 expression was significantly increased in the OE-RP11-815M8.1 group compared with the pBABE group. (b) The expression of lncRNA RP11-815M8.1 in the sh-RP11-815M8.1 group was significantly decreased compared with that in the PLKO.1 group (^∗^*p* < 0.05, ^∗∗^*p* < 0.01).

**Figure 3:** Effects of the overexpression and knockdown of lncRNA RP11-815M8.1 on hBMSC growth (^∗^*p* < 0.05, ^∗∗^*p* < 0.01).

**Figure 4:** Alizarin red staining results 14 days after osteogenic differentiation of hBMSCs transfected with lentiviral vectors for the overexpression and knockdown of lncRNA RP11-815M8.1. hBMSCs transfected with the lncRNA RP11-815M8.1-overexpressing lentiviral vector (OE-RP11-815M8.1 group), lncRNA RP11-815M8.1-knockdown lentiviral vector (sh-RP11-815M8.1 group), and the corresponding empty transfection vector controls (pBABE group, PLKO.1 group).

**Figure 5:** Expression of osteogenic transcription factors. (a) Expression of osteogenic transcription factors in hBMSCs transfected with the lncRNA RP11-815M8.1-overexpressing lentiviral vector 14 days after osteogenic differentiation. (b) Expression of osteoblastic-specific transcription factors in hBMSCs transfected with lncRNA RP11-815M8.1-knockdown lentiviral vectors 14 days after osteogenic differentiation (^∗^*p* < 0.05, ^∗∗^*p* < 0.01).

**Figure 6:** Correlation network diagram of lncRNAs, miRNAs, and mRNAs. In the figure, lncRNAs are represented in red, mRNAs are represented in brown, and miRNAs are represented in green.

**Table 1:** Gene sequences of lncRNA RP11-815M8.1.

Gene name	Official symbol	Gene sequences
RP11-815M8.1	LINC02257	AGATGCACATGAAATTTGGTGCCGTGACTCGGATTGGGGGACCTCCCTTGGGAGATCAATCCCCTGTACTCCTGTTCTTTGCTCCGTGAGAAAGATCCACCTATGACCCTCAGGTCCTCAGACCGACTAGCCCAAGGAACATCTCACCAATTTTAAATCAGGTGGAGTCTCGCACTGTCATCCTGGCTGGAATGCAGTGGTGCAAGCCGACTCACTGCAACCTCTGCCTCTTGGGTTCAAGTGATTCTCCTGCTTCAGCCTCCTGATTTGCTGGGATTGCAGAGCAAACCAGTGAAAAAATGGCCTTCGCACTCCTGAGAGACCTTTCACCGGGCTTTCTACTTTTGAATTCTCTCCATAGCTGGTTTCCTCTTAGGCCTCGATAGAGCAGTCCCTGAATCACACAGGTATGCTGACTACGTCTTTTCCTGGTACAAACCATCATGGGGGAAACACACAGCAAGAAGCATCTTCAGGTCACAAGATAGGTAATACCATCTACCTGAATTTTTTCAAAAGCAGCAGAATATTTAGTTTTCTATTTCAGTGGCTTCTAACAGAGATCATTGTTTGCACAAGATTAAATGTCTGCAGTGGTCGTCTTAAAAAAAAA

**Table 2:** Sequences of primers for RT-PCR.

Primer	Primer sequence (5′-3′)
h-lncRNA RP11-815M8.1 qF	CTAGCCCAAGGAACATCTCAC
h-lncRNA RP11-815M8.1 qR	AGCAGGAGAATCACTTGAACC
h-ALP qF	AGAATCTGGTGCAGGAATGG
h-ALP qR	TCGTATTTCATGTCTCCAGGC
h-OCN qF	TGCAGCCTTTGTGTCCAAG
h-OCN qR	CCCAGCCATTGATACAGGTAG
h-OPN qF	AGGCTGATTCTGGAAGTTCTG
h-OPN qR	CTTACTTGGAAGGGTCTGTGG
h-Runx2 qF	TTCACCTTGACCATAACCGTC
h-Runx2 qR	GGCGGTCAGAGAACAAACTAG
h-Osterix qF	CCACCTACCCATCTGACTTTG
h-Osterix qR	CCACTATTTCCCACTGCCTT
h-GAPDH qF	TGTTGCCATCAATGACCCCTT
h-GAPDH qR	CTCCACGACGTACTCAGCG

**Table 3:** Changes in the expression level of lncRNA RP11-815M8.1 before and after osteogenic differentiation of hBMSCs.

lncRNA	D0	D7	D14	D21
RP11-815M8.1	1.01 ± 0.20	22.31 ± 2.74	39.51 ± 3.72	59.39 ± 1.67

**Table 4:** Efficiency of lentiviral vector transfection for the overexpression and knockdown of lncRNA RP11-815M8.1.

lncRNA	pBABE	OE-RP11-815M8.1	PLKO.1	sh-RP11-815M8.1
RP11-815M8.1	1.39 ± 1.41	55.90 ± 9.40	1.05 ± 0.36	0.11 ± 0.10

**Table 5:** Expression of osteogenic transcription factors in hBMSCs transfected with the lncRNA RP11-815M8.1-overexpressing lentiviral vector 14 days after osteogenic differentiation.

Osteogenic transcription factors	D0	D14
ALP	1.04 ± 0.35	3.89 ± 0.67
OCN	1.00 ± 0.04	2.27 ± 0.10
OPN	1.00 ± 0.11	2.51 ± 0.06
Runx2	1.00 ± 0.06	3.74 ± 0.87
Osterix	1.01 ± 0.19	4.79 ± 0.66

**Table 6:** Expression of osteogenic transcription factors in hBMSCs transfected with the lncRNA RP11-815M8.1-knockdown lentiviral vector 14 days after osteogenic differentiation.

Osteogenic transcription factors	D0	D14
ALP	1.02 ± 0.25	0.27 ± 0.02
OCN	1.00 ± 0.05	0.38 ± 0.15
OPN	1.00 ± 0.05	0.36 ± 0.01
Runx2	1.00 ± 0.09	0.33 ± 0.09
Osterix	1.01 ± 0.19	0.24 ± 0.05

## Data Availability

The data used to support the findings of this study are available from the first author upon request.
